The article "Cytotoxicity and Genotoxicity of Biogenic Silver Nanoparticles in A549 and BEAS-2B Cell Lines" was published in 2022. Journal: Bioinorg Chem Appl.

# Cytotoxicity and Genotoxicity of Biogenic Silver Nanoparticles in A549 and BEAS-2B Cell Lines

**DOI:** 10.1155/2022/8546079

**Published:** 2022-09-23

**Authors:** Musthahimah Muhamad, Nurhidayah Ab.Rahim, Wan Adnan Wan Omar, Nik Nur Syazni Nik Mohamed Kamal

**Affiliations:** ^1^Department of Toxicology, Advanced Medical and Dental Institute, Universiti Sains Malaysia, 13200 Kepala Batas, Penang, Malaysia; ^2^Department of Medical Laboratory Technology, Faculty of Health Sciences, Universiti Teknologi MARA, 13200 Kepala Batas, Penang, Malaysia

## Abstract

**Introduction:**

Biogenic silver nanoparticles (AgNPs-GA) were successfully synthesised using *Garcinia atroviridis* leaf extract as a reducing agent, which has ethnopharmacological claims against various diseases including cancer. *Aim of the Study*. Aim of the study is to discover whether AgNPs-GA has cytotoxic and genotoxic effects on cancerous (A549) and noncancerous (BEAS-2B) human lung cells.

**Materials and Methods:**

The cytotoxicity profiles of AgNPs-GA were characterized by MTT assay, intracellular reactive oxygen species (ROS) assay, and DAPI and AOPI double staining, whilst genotoxicity was assessed using Comet Assay analysis. The level of silver ions (Ag^+^) and cellular uptake of AgNPs-GA were evaluated by ICP-OES and TEM analyses, respectively.

**Results:**

A significant cytotoxic effect was observed by AgNPs-GA on both A549 and BEAS-2B cell lines, with IC_50_ values of 20–28 *μ*g/ml and 12–35 *μ*g/ml, respectively. The cytotoxicity profile of AgNPs-GA was also accompanied by a pronounced increase in ROS production, DNA damage, and apoptosis. Moreover, Ag^+^ was also detected in cells exposed to AgNPs-GA threefold higher compared to controls. In this study, AgNPs-GA were endocytosed within lysosomes, which may direct to secondary toxicity effects including oxidative stress, impairment of the cell membrane, DNA fragmentation, and cell death.

**Conclusions:**

Taken together, novel toxicological-related mechanisms by AgNPs-GA were proposed involving the generation of ROS that causes DNA damage which led to programmed cell death in both A549 and BEAS-2B cells. Therefore, a combination of scientific assessments is constantly needed to ensure that the quality of biosynthesized nanoparticles is controlled and their safe development is promoted.

## 1. Introduction

Nanotechnology covers the study and application of matter at the nanoscale between 1 and 100 nanometers (1 nm = 10^−9^ m) [1]. It is among the most widely used technologies in translational research. Objects at this scale, such as “nanoparticles,” hold many potential applications in clinical medicine and research, such as delivering drugs more effectively, diagnosing diseases more rapidly and sensitively, and treating diseases efficiently [2]. In the field of nanotechnology, metallic nanoparticles (MNPs) are widely utilised in biomedical sciences and engineering. For example, MNPs serve a good candidate for wound dressing materials as well as desirable materials used in the biosensor interface design [3]. Their high surface to volume ratio and high reactivity are described to influence the aforementioned potential and wider applicability [3]. Among several metallic nanoparticles, silver nanoparticles (AgNPs) are the inorganic metal-based choice as they possess attractive physicochemical properties and biological functionality. There are several methods for synthesising AgNPs, including physical, chemical, and biological procedures [1, 4]. Emphasis has been given to the production of AgNPs that confers a simple, value-effective, and environment-friendly technique, in keeping with global efforts to reduce generation of hazardous waste and high energy consumption [5]. This is because the use of toxic solvents and chemical contamination could exert potential hazards including carcinogenicity, toxicity, and environmental toxicity [6]. For these reasons, AgNPs made by green synthesis technology offer a novel, eco-friendly, and sustainable procedure to overcome the aforementioned shortcomings [7]. Nonetheless, AgNPs produced through green synthesis route should follow three requirements as stated in the green chemistry dogma. These include a combination of a biocompatible and nontoxic solvent medium, environmentally benign reducing agents, and nontoxic substances for stabilization of the nanoparticles [5].

The article "Cytotoxicity and Genotoxicity of Biogenic Silver Nanoparticles in A549 and BEAS-2B Cell Lines" was published in 2022. Journal: Bioinorg Chem Appl.

There are two common strategies in use for the synthesis of inorganic nanoparticles, namely, the top-down approach and the bottom-up approach [4]. The top-down approach involves the breaking down of the bulk material into nanosized structures or particles, wherein it is usually carried out by physical, chemical, or mechanical processes [8]. On the contrary, the bottom-up approach uses chemical or physical forces or biological resources to assemble basic units such as molecules or atoms in order to build up nanoparticles [9]. The major advantage of chemical synthesis is high-yield production of AgNPs. Chemical reduction using different types of organic and inorganic reducing agents, electrochemical techniques, physicochemical reduction, and radiolysis are the most commonly applied methods for the production of AgNPs [10]. However, the abovementioned techniques involve the use of hazardous chemicals that may result in toxic byproducts and environmental toxicity [11, 12]. Apart from these drawbacks, some key issues such as stability, aggregation, and purity of nanoparticles may limit the quality and quantity of the synthesised nanoparticles for further applications [10, 12]. Through physical processes, AgNPs are commonly synthesised by evaporation-condensation and laser ablation methods [10, 12, 13]. The physical route renders several advantages including speed, and the use of radiation as reducing agents could reduce the need of using hazardous chemicals [12, 13]. However, synthesis of AgNPs via physical route usually gives small number of AgNPs in contrast with chemical process [14]. Additionally, physical synthesis of AgNPs occupies a large space to accommodate tube furnace and other related instruments, requires long duration for completion of the whole process, and utilises high energy consumption over the long run that may lead to an excessive heat to surroundings [10, 13].

The article "Cytotoxicity and Genotoxicity of Biogenic Silver Nanoparticles in A549 and BEAS-2B Cell Lines" was published in 2022. Journal: Bioinorg Chem Appl.

To address the abovementioned issues, alternative route for AgNPs production through green chemistry including the use of biological sources has demonstrated superiorities over conventional chemical and physical synthesis. In this regard, green synthesis of AgNPs has several merits; for example, it is simple, rapid, and inexpensive, with plethora of choices and accessible amounts of resources, biocompatibility, and easy procedures to control and optimize well-defined size and morphology, produces high yield, solubility, and stability of AgNPs, requires less time consumption, is environment-friendly as it uses nontoxic chemicals, and is easily scaled up for large scale applications [9, 15–18].

It is important to note here that living system has the ability to transform metallic ions into nanoparticles by manipulating its intrinsic organic chemistry processes [4]. In this regard, biological systems such as plants [19], fungi [20], bacteria [21], algae [22], seaweed [23], lichen [24], and small biomolecules including amino acids, proteins, enzymes, and carbohydrates [9, 12] have been broadly researched for the production of AgNPs. Among the aforesaid bioresources, synthesis of AgNPs using plant (inactivated plant tissue, plant extracts, and living plant) has become an important branch of biosynthesis processes [17]. This may be owing to the ability of plants to produce a wide array of secondary metabolites such as sugars, alkaloids, phenolic acids, terpenoids, and polyphenols, with strong reducing potential [25]. In this context, Fourier transform infrared (FTIR) is routinely performed to identify the functional groups involved in the formation of AgNPs [26]. For example, according to this characterization, the difference in the FTIR spectra between green tea leaf extract (GT) and GT AgNPs was used to indicate the functional groups involved in the reduction of silver salts into nanoparticles [26]. In addition to these, plant-mediated green synthesis of nanoparticles is easy to scale up due to the availability of plant products, being environment- and economy-friendly, that further justify its outstanding applications in various fields [18, 27]. Moreover, plants are preferred over microbes because they are nonpathogenic. Thus, it can be considered safe to be employed in the pharmaceutical, biomedical, and food industries [4].

The article "Cytotoxicity and Genotoxicity of Biogenic Silver Nanoparticles in A549 and BEAS-2B Cell Lines" was published in 2022. Journal: Bioinorg Chem Appl.

The application of nanomedicine in pharmaceutical and biotechnology industries has seen profound effects. In this regard, currently about 50 to 100 nanomedicine formulations and nano-based pharmaceutical products have been approved for clinical use including drug delivery, bioimaging, biomaterials, and diagnostic or other medical devices [1, 28, 29]. Through nanotechnology, nanomaterials including AgNPs have been developed as an important strategy to deliver conventional drugs, recombinant proteins, vaccines, and nucleotides [2]. Besides, owing to their antimicrobial properties, such nanoparticles are integrated in various materials of everyday use such as toothpaste, water purification systems, and humidifiers [4]. As described by the authors [4], plant-mediated AgNPs are also effective against diverse Gram-negative and Gram-positive agricultural pathogens. Apart from the abovementioned properties, AgNPs also exhibit an antitumorigenic ability due to their cytotoxicity against various tumor models [30]. For example, AgNPs produced by *Catharanthus roseus* leaf extract exhibited anticancer effect by suppressing growth, migration, and invasion of HepG2 human hepatocellular carcinoma cells *in vitro* [31].

Malaysia is recognized as a country that is rich in the medicinal plant species, which are regarded as preeminent sources of substances that can be used for therapeutic and pharmaceutic purposes [32, 33]. Among them is *Garcinia atroviridis* (*G. atroviridis*), an edible and seasonal fruit tree that is traditionally used for cough, throat irritation, earache, and pre- and postpartum medication [34, 35]. The fruits and leaves of this plant are locally consumed among Malay and indigenous communities as flavouring agent and salads [34, 35]. As abovementioned, biosynthesized AgNPs are regarded as green products; however, toxicological status and nanosafety of these bioengineered nanomaterials are poorly understood or rather unclear. Therefore, the aim of the present study was to evaluate the mechanisms of toxicity and explore possible risks associated with bioengineered AgNPs. To the best of our knowledge, there is no particular study of toxicological profiles of biosynthesized AgNPs from *G. atroviridis* leaf extract against human lung cell model. Thus, the novelty of study presented herein lies on the new data of nanotoxicity, nanogenotoxicity, and cytotoxicological pathways involved following exposure to the biosynthesized AgNPs-GA on A549 and BEAS-2B human lung cell model.

The article "Cytotoxicity and Genotoxicity of Biogenic Silver Nanoparticles in A549 and BEAS-2B Cell Lines" was published in 2022. Journal: Bioinorg Chem Appl.

## 2. Materials and Methods

### 2.1. Preparation of Plant Extract

*G. atroviridis* leaves were collected from Kepala Batas, Penang, Malaysia. The herbarium of Universiti Sains Malaysia, Penang, Malaysia, has been deposited with a voucher specimen (11764). The fresh leaves were washed, and the particles were removed with clean water. The leaves were then dried in an industrial hot air oven at 40°C for three days and ground with a herb grinder.

### 2.2. Biosynthesis of Silver Nanoparticles (AgNPs-GA)

AgNPs-GA were synthesised using our previously described process [36]. Briefly, the optimal concentration of *G. atroviridis* used in this analysis was 10% of the leaf extract and 0.1 M of aqueous AgNO_3_ (Nacalai Tesque Chemicals, Kyoto, Japan) that were mixed at a ratio of 1 : 4. The optimum reaction time was calculated for the incubation period from 24 to 72 hours at 32°C. Colour changes of the reaction mixture from light yellow to dark brown were observed. The bioreduction of silver ions in the solution was then periodically monitored by the absorption peak at 400–450 nm in the UV-visible spectrum. The pH of the reaction mixture was calculated to maximise the yield and properties of AgNPs-GA. The samples were purified, freeze-dried, and stored for further analysis. The AgNPs-GA were characterized using FTIR, TEM, SEM, zeta potential, Dynamic Light Scattering (DLS), and XRD as reported in our previous study [36].

### 2.3. Cell Culture

The cytotoxic effect of AgNPs-GA, AgNPs (commercial), *G. atroviridis* aqueous extract (Leaf-GA), and silver nitrate (AgNO_3_) on A549 and BEAS-2B cells were assessed. Both A549 and BEAS-2B cells were originally purchased from the American Type Culture Collection (ATCC, USA). Both cells were cultured in Dulbecco's Modified Eagle's Medium (DMEM: Gibco, USA) and 1 : 1 mixture of DMEM and Ham's F-12 (DMEM-F12; Gibco, USA) medium with phenol red and supplemented with 10% fetal bovine serum (FBS; Gibco, USA), 0.1% (v/v) penicillin-streptomycin, and 2 mM L-glutamine (PenStrep; Gibco, USA). The cell lines were maintained in a humidified environment at 37°C with 5% CO_2_.

The stock solution of AgNPs-GA, AgNPs (commercial), Leaf-GA, and AgNO_3_ was prepared to a final concentration of 10 mg/mL and stored at −20°C until further analysis. The Cisplatin stock solution (5 mg/ml or 1.67 mM with a purity of approximately 98.0% (T); Merck, Germany) was prepared in 0.9% sodium chloride (NaCl) and stored at −20°C until further use.

The article "Cytotoxicity and Genotoxicity of Biogenic Silver Nanoparticles in A549 and BEAS-2B Cell Lines" was published in 2022. Journal: Bioinorg Chem Appl.

### 2.4. 3-(4,5-Dimethylthiazol-2-yl)-2,5-Diphenyltetrazolium Bromide (MTT) Assay

The cytotoxicity effects of AgNPs-GA, AgNPs (commercial), Leaf-GA, and AgNO_3_ against A549 and BEAS-2B cells were evaluated using a typical colorimetric (3-(4,5-dimethylthiazol-2-yl)-2,5-diphenyltetrazolium bromide (MTT)) proliferation assay (Sigma-Aldrich, St. Louis, Missouri, USA). The adhered cells were incubated at 37°C for 24–72 hours with culture medium only (untreated cells or negative control) and fresh assay medium treatments complemented with increasing concentrations of 10–100 *μ*g/mL of AgNPs-GA, AgNPs (commercial), Leaf-GA, and (10–100 *μ*M) AgNO_3_. The culture medium alone (without cells) was included as a blank for this test. A549 and BEAS-2B cells were treated with Cisplatin as a positive control. A total of 10 *μ*L of MTT solution (5 mg/mL) was applied to each well at about 24 to 72 hours after treatment and was further incubated for 4 hours in the dark at 37°C with 5% CO_2_. Upon incubation, the mixture solution was aspirated, and 100 *μ*L of dimethyl sulfoxide (DMSO) (Fisher Scientific, USA) was added to solubilise the purple formazan. The optical density (O.D.) of each sample was measured at a 570 nm wavelength using a microplate reader (BioTek Instruments, Inc, USA). The percentage (%) of cell viability was determined using the following formula [37]:

(1) $$\begin{array}{c} \text{Cell viability}\left(\text{\%}\right)=\frac{\text{O.D.treatment–O.D.blank}}{\text{O.D.untreated cell–O.D.blank}}\times 100\text{\%.} \end{array}$$

Based on the measured cell viability (%), a graph was created to display the dose-response curves for each cell line. The IC_50_ values for each treatment, which affect 50% of cell viability, were calculated from this graph at 50% cell viability. The data was expressed as a mean and standard deviation with each experiment consisting of triplicates. Statistical differences between untreated cells and treated cells were determined using Student's *t*-test (IBM SPSS Statistics 27).

#### 2.4.1. Selectivity Index (SI)

The degree of selectivity of AgNPs-GA, AgNPs (commercial), Leaf-GA, and AgNO_3_ towards cancer cells can be expressed by the selectivity index (SI) value [38], which was calculated using the formula as follows:

(2) $$\begin{array}{c} \text{Selectivity index}\left(\text{SI}\right)=\frac{\text{IC}50\text{ normal cells}}{\text{IC}50\text{ cancer cells}}. \end{array}$$

### 2.5. Detection of ROS Production by 5-(and-6)-Chloromethyl-2′,7′-Dichlorodihydrofluorescein Diacetate, Acetyl Ester (CM-H2DCFDA) Assay

Following the manufacturer's guidelines, the generation of intracellular ROS using a 5-(and-6)-chloromethyl-2′,7′-dichlorodihydrofluorescein diacetate, acetyl ester (CM-H2DCFDA) detection reagents (Invitrogen, Thermo Fisher Scientific, USA) was determined. Briefly, A549 and BEAS-2B cells were seeded in 96-well plates and treated for 24 hours with IC_50_ of AgNPs-GA, Cisplatin, and a combination of AgNPs-GA + Cisplatin. After exposure, cells were washed with PBS and loaded with 2.5 *μ*M of CM-H_2_DCFDA in phenol red and FBS-free media in the dark for 30 minutes at 37°C. Subsequently, the reaction mixture was aspirated; cells were washed with fresh culture media and replaced with 100 *μ*L of culture media. The DCF fluorescence intensity was measured at 485 nm excitation and 520 nm emission using a FLUOstar Omega fluorescence plate reader (BMG Labtech, Ortenberg, Germany). Results are presented as mean fold change ± standard deviation of three independent experiments.

The article "Cytotoxicity and Genotoxicity of Biogenic Silver Nanoparticles in A549 and BEAS-2B Cell Lines" was published in 2022. Journal: Bioinorg Chem Appl.

### 2.6. DNA Damage Analysis

The Comet Assay® kit (Trevigen, Inc, USA) was used to perform DNA damage activity analysis. Cells were seeded into T25 flasks at a density of 5 × 10^5^ cells and treated with respective IC_50_ of AgNPs-GA, Cisplatin, and a combination of AgNPs-GA + Cisplatin for 24 hours. Following this, cells were treated with 100 *μ*M of H_2_O_2_ for 20 minutes. After being detached by Accutase (BD™Bioscience, USA), the cells were collected and washed with ice-cold PBS. According to the manufacturer's protocol, the cell pellets were mixed in a ratio of 1 : 10 (v: v) with a low melting point agarose and pipetted onto CometSlide™. The cells were then lysed in the lysis solution at 4°C for 30 minutes. Then, the cells were kept in an alkaline unwinding solution at room temperature for 20 minutes to allow the DNA to unwind. The test was immediately followed by electrophoresis, performed at 21 V and 300 mA for 30 minutes. Slides were washed in 70% ethanol and water and stained with SYBR® gold nucleic acid gel stain (Invitrogen, Thermo Fisher Scientific, USA) before visualisation under the Olympus IX71 inverted fluorescence microscope (Olympus, Tokyo, Japan). A total of 50 cells were randomly selected and captured per sample at 100× magnification and analysed using the Open Comet Image J available at https:/www.cometbio.org/. Tail length, percentage of tail DNA, and Olive Tail Moment (OTM) were calculated for DNA damage assessment.

### 2.7. Mechanism of Apoptosis by DAPI and Acridine Orange (AO) and Propidium Iodide (PI) Double Staining

DAPI staining is used to assess apoptosis-related morphological changes such as nuclear fragmentation or condensation. The acridine orange/propidium iodide stain used in dual staining shows the apoptotic induction caused by the AgNPs treatment. AO stains both live and dead cells, whereas PI stains only the dead cells. In brief, 3 × 10^5^ of both A549 and BEAS-2B cells were seeded separately in the 6-well plates and treated with appropriate IC_50_ values of AgNPs-GA, Cisplatin, and AgNPs-GA + Cisplatin for 24 hours at 37°C with 5% CO_2_. Following incubation, the cells were washed with PBS and then fixed with 1 mL of 4% paraformaldehyde (Sigma-Aldrich, St. Louis, Missouri, USA) and cold 70% ethanol for 10 minutes at room temperature. Then, the cells were stained with a 1 : 1 ratio of 10 *µ*g/mL of DAPI (Nacalai, Tesque chemical, Kyoto, Japan) and 10 *μ*g/mL acridine orange/propidium iodide (Sigma-Aldrich, St. Louis, Missouri, USA) and incubated for 30 minutes in the dark. An Olympus IX71 inverted fluorescence microscope (Olympus, Tokyo, Japan) was used to observe and record the morphology of the cells.

The article "Cytotoxicity and Genotoxicity of Biogenic Silver Nanoparticles in A549 and BEAS-2B Cell Lines" was published in 2022. Journal: Bioinorg Chem Appl.

### 2.8. Measurement of Intracellular Ag^+^ and Cellular Uptake of AgNPs

The intracellular Ag^+^ concentration and uptake of AgNPs-GA, Cisplatin, and AgNPs-GA + Cisplatin in the A549 and BEAS-2B cells were analysed by inductively coupled optical emission spectroscopy (ICP-OES) and visualised using TEM. The cells were seeded in a T75 cell culture flask at a density of 3 × 10^6^ cells per ml growth medium and exposed to IC_50_ values of AgNPs-GA, Cisplatin, and AgNPs-GA + Cisplatin. Control cells were incubated in a standard cell medium (DMEM supplemented with 10% FBS and antibiotics). After a treatment period of 24 hours, the cells were harvested using 0.25% enzyme trypsin, then washed with PBS (pH 7.4), collected, and centrifuged at 1500*g* for 10 min at 4°C. The cell pellets were further evaluated for ICP-OES and TEM analysis.

#### 2.8.1. Inductively Coupled Plasmon Optical Emission Spectroscopy (ICP-OES)

Silver concentrations in the digested samples were measured using an Agilent Technologies 700 series ICP-OES (Agilent, Waldbronn, Germany). Briefly, the cell pellets were digested in a 5 ml solution of 65% HNO_3_. Digestion was performed in closed vials at 60°C using a heating block for 30 hours. Then, the digested sample was made up to 50 mL with ultrapure water (18.2 MΩcm) (GenPure UV; TKA) and kept at 4°C until further use. Calibrations were performed using silver standard (1000 ppm in ca. M HNO_3_ solution) (Fisher Scientific, USA) with measurements ranging from 0 to 2 ppm. Every experiment was conducted in three independent replicates for each treatment and control group.

#### 2.8.2. Transmission Electron Microscopy (TEM)

In general, the cell pellets were fixed in McDowell-Trump fixative (overnight) and then post-fixed with 1% osmium tetraoxide for 1 hour at room temperature. Subsequently, the cells were washed thoroughly and dehydrated using a series of graded ethanol (50%, 70%, and 95%) for 15 minutes each and 30 minutes, respectively in 100% ethanol. Cells were further dehydrated using 100% acetone for 10 minutes, followed by overnight infiltration with acetone using Spurr's resin mixture (1 : 1). The cells were then further penetrated with a fresh change of pure Spurr's resin for 3 days and finally embedded in pure Spurr's resin at 60°C in an oven overnight. The specimen blocks were ultrathin sectioned on a PowerTomeXL ultramicrotome (RMC Boeckeler Instruments, Inc., Tucson, Arizona, USA) using a knife-boat and an Ultra 45 Diatome diamond knife (Diatome, Biel, Switzerland) with 70–90 nm per section. The sections were collected on copper grids and stained with uranyl acetate and lead citrate for imaging using energy-filtered transmission electron microscopy (EFTEM) Libra 120 (Carl Zeiss Meditec AG, Jena, Germany).

The article "Cytotoxicity and Genotoxicity of Biogenic Silver Nanoparticles in A549 and BEAS-2B Cell Lines" was published in 2022. Journal: Bioinorg Chem Appl.

### 2.9. Statistical Analysis

The data was presented as a mean and standard deviation (mean ± SD). All the *in vitro* studies involved three independent experiments, with each experiment consisting of three replicate measurements. SPSS Statistics 27 (IBM, USA) was used to analyse statistical differences between untreated cells and treated cells using Student's *t*-test. For the multiple comparison test, one-way analysis of variance (ANOVA) was used, followed by a post hoc Turkey. *P* < 0.05 was considered statistically significant.

## 3. Results

### 3.1. Biosynthesis of Silver Nanoparticles Mediated *G. atroviridis* Leaves Extract

AgNPs-GA biosynthesis was formed using 10% (w/v) Leaf-GA and 0.1 M AgNO_3_ solution at a ratio of 1 : 4 at 32°C. The light brown colour of the Leaf-GA was transformed into a dark brown solution due to silver plasmon resonance formation (Figure 1(a)) and Ag^+^ions to Ag^o^ by the Leaf-GAs [39]. Based on the UV-visible spectroscopy, the maximum absorption of AgNPs-GA was at 440–450 nm at pH 3.02 compared to the Leaf-GA and 0.1 M AgNO_3_ solution alone. The broadening peak was observed indicating that the particles polydispersed. The synthesis of AgNPs-GA increased with an increasing incubation time of the Leaf-GA along with the AgNO_3_ solution at 24, 48, and 72 hours (Figure 1(b)). This could be due to increased formation or agglomeration of AgNPs-GA. This finding is consistent with another study that concluded small-sized metal nanoparticles formed at pH 3.0 and 4.0 would bind to many functional groups and nucleate metal ions [40].

The article "Cytotoxicity and Genotoxicity of Biogenic Silver Nanoparticles in A549 and BEAS-2B Cell Lines" was published in 2022. Journal: Bioinorg Chem Appl.

The physicochemical characteristics of AgNPs-GA were previously described by our group in [36]. SEM analysis indicated that AgNPs-GA morphology was spherical and it was aggregated as clusters. This finding was further supported by TEM analysis that demonstrated the shape of AgNPs-GA formed is predominantly spherical and 5–30 nm in size. The average hydrodynamic diameter (*Z*-average) of AgNPs-GA was 176 nm and zeta potential of nanoparticles was −24.4 mV. The *Z*-average of AgNPs-GA was reasonably higher than its TEM-assessed particle diameters, which suggests our nanomaterials were more susceptible towards aggregation. In addition, polydispersity index (PDI) value of AgNPs was 0.4, indicating that AgNPs-GA has good dispersity, in between monodispersed and polydispersed, and is metastable. The XRD spectrum revealed four prominent diffraction peaks at 2*θ* values of 38.12°, 44.20°, 64.68°, and 77.55°, in the range of 30–70° at 2*θ* angles, which correspond to (111), (200), (220), and (311) Bragg's reflection planes of metallic silver's faced-centered cubic (fcc) structure. The average particle size of AgNPs-GA was calculated using the Debye-Scherrer equation and was found to be 14.64 nm. The FTIR spectrum for *G. atroviridis* leaf extract showed the absorption bands at 1030 cm^−1^ (-C-O stretching), 1622 cm^−1^ (-C=C-stretching), 1728 cm^−1^ (-C=O stretching), 2920 cm^−1^ and 2851 cm^−1^ (-CH stretching), and 3332 cm^−1^ (-OH stretching), as described in our previous report [36]. The observed bands suggest the occurrence of flavonoids and phenolic compounds in the *G. atroviridis* leaf extract. In AgNPs-GA, the peak shifted, suggesting the effect of these functional groups of *G. atroviridis* leaf extract as reducing and stabilizing agents in mediating the biosynthesis of AgNPs-GA.

### 3.2. In Vitro Assessment of AgNPs-GA, Leaf-GA, AgNO_3_, and AgNPs (Commercial) Toxicity on A549 and BEAS-2B Cell's Viability

Growth inhibitory effects of AgNPs-GA, Leaf-GA, AgNO_3_, and AgNPs (commercial) treatments on A549 and BEAS-2B cells are shown in Figures 2(a) and 2(b), respectively. Viable cells that have active metabolism will transform MTT into a coloured, purple formazan substance with a 570 nm absorbance value. In contrast, dead cells lose their capability to change MTT to formazan [41]. In this study, after 24 to 72 hours of treatment, AgNPs-GA at 30–100 *μ*g/mL reduced the proliferation of A549 cells (Figure 2(a) (i)) to 50% or more by 24 hours. However, AgNPs-GA were toxic to BEAS-2B cells (Figure 2(b) (i)) where more than 50% of cell death was observed at a concentration of 40–100 *μ*g/mL (treatment for 24 hours) and 20–100 *μ*g/mL (treatment for 72 hours). AgNPs-GA, which are proven to have a potent antiproliferative effect on A549 cells, were also toxic to BEAS-2B cells.

The article "Cytotoxicity and Genotoxicity of Biogenic Silver Nanoparticles in A549 and BEAS-2B Cell Lines" was published in 2022. Journal: Bioinorg Chem Appl.

In this study, the Leaf-GA showed weak cytotoxicity effect to both A549 (Figure 2(a) (ii)) and BEAS-2B (Figure 2(b) (ii)) cells at a concentration of 65 to 350 *μ*g/ml (24 to 72 hours). As a result, a higher dosage of crude extract was required to induce cytotoxicity.

Moreover, AgNO_3_ decreases the proliferation of both A549 (Figure 2(a) (iii)) and BEAS-2B (Figure 2(b) (iii)) cells to nearly 50% after 24 to 74 hours of treatment with concentrations of 40–100 *μ*M and 20–100 *μ*M, respectively. However, AgNO_3_ displayed cytotoxicity activity towards the cells. The reduction of silver ions in the biosynthesised AgNPs-GA demonstrated potential antiproliferative properties.

AgNPs (commercial) are defined as silver <100 nm containing polyvinylpyrrolidone (PVP) as a dispersant. AgNPs (commercial) demonstrated dose-dependent cell death by more than 50% over time. AgNPs (commercial) showed weak cytotoxicity activity against both A549 and BEAS-2B cells at 24 hours after treatment (Figures 2(a) (iv) and 2(b) (iv)). As a result, a higher dosage of AgNPs (commercial) and longer incubation period were needed to exhibit antiproliferative effect.

In comparison, both A549 and BEAS-2B were significantly dead at 50 *μ*M and 65 *μ*M Cisplatin (the standard chemotherapy agent for lung cancer) at all three time points tested in this analysis.  Table 1 summarises the average IC_50_ profiles of AgNPs-GA, Leaf-GA, AgNO_3_, and AgNPs (commercial) against A549 and BEAS-2B cell lines, as well as the SI.

SI is determined by comparing the IC_50_ of the normal cells to the IC_50_ of the cancer cells [38]. A higher SI value (>2) suggests that the extracts or compounds produce selective toxicity towards cancer cells. A lower SI value (<2) is considered general toxicity, in which it also can cause cytotoxicity in normal cells [42].

SI values of AgNPs-GA, Leaf-GA, AgNO_3_, and AgNPs (commercial) were less than twofold cytotoxic selectivity in A549 cells (Table 1). This value means that the aforementioned treatments possess comparable cytotoxic effect to both A549 cancer and BEAS-2B normal cell lines. These SI values also indicate that the tested cytotoxic agents possess general toxicity rather than selective toxicity. In this regard, treatment with these cytotoxic agents is worth further investigation to understand possible underlying mechanism of its general toxicity.

### 3.3. Analysis of Reactive Oxygen Species (ROS) Generation

The potential of AgNPs-GA, Cisplatin, and AgNPs-GA + Cisplatin to induce oxidative stress was assessed using the CM-H2DCFH-DA assay by measuring the intracellular ROS levels. During the treatment, an increase in ROS formation was observed in A549 and BEAS-2B cells demonstrated by an increase of DCF fluorescence intensity. As seen in Figure 3 and compared to the control, significantly increased ROS levels were observed, indicated by DCF fold with AgNPs-GA (1.25 ± 0.02), Cisplatin (1.16 ± 0.04), and the combination of AgNPs-GA + Cisplatin (1.23 ± 0.09) treated A549. Meanwhile, BEAS-2B exhibited higher ROS levels treated with AgNPs-GA (1.28 ± 0.02), Cisplatin (1.23 ± 0.01), and the combination of AgNPs-GA + Cisplatin (1.29 ± 0.05), respectively.

The article "Cytotoxicity and Genotoxicity of Biogenic Silver Nanoparticles in A549 and BEAS-2B Cell Lines" was published in 2022. Journal: Bioinorg Chem Appl.

### 3.4. Analysis of DNA Damage Activity

DNA damage activity was assessed using Comet Assay analysis or also known as Single Cell Gel Electrophoresis (SCGE), which is utilised to determine the amount of DNA damage in a single cell. Additionally, both A549 cells and BEAS-2B cells were damaged due to the treatment with AgNPs-GA, Cisplatin, AgNPs-GA + Cisplatin, and H_2_O_2_ using the Comet Assay.  Table 2 represents the tail length (px), percentage of DNA in the tail, and OTM as the relevant parameters to investigate both untreated cells and treated cells. Cisplatin, a chemotherapeutic, and H_2_O_2_, an oxidant, were both used as positive controls.

Figures 4 and 5 demonstrate that treatment with AgNPs-GA enhances DNA damage to Class 4 against A549 cells. Collins and colleague [43] suggested the images of comet into Classes 0–4 to be used for visual scoring. The increased number of classes represents the increase in DNA damage severity.  Figure 4 demonstrates the morphological changes in untreated and treated A549 and BEAS-2B cells. There was a significant Class 3 DNA damage found in Cisplatin treatment and the combination of AgNPs-GA + Cisplatin against A549 cells. Class 2 DNA damage was also observed in A549 cells treated with 100 *μ*M of H_2_O_2_ (Figure 4(a)). DNA percentage (%) in the tail of untreated, AgNPs-GA, Cisplatin, AgNPs-GA + Cisplatin, and H_2_O_2_ was 2.05 ± 0.37, 87.9 ± 3.96, 48.26 ± 4.54, 59.2 ± 1.6, and 35.64 ± 9.31, respectively (Table 2) (Figure 5(a)). Tail length is used to determine the extent of DNA damage as it is the distance of DNA migration from the nuclear core body. Tail-length products and the total DNA fractions in the tail define the OTM [44]. The untreated, AgNPs-GA, Cisplatin, AgNPs-GA + Cisplatin, and H_2_O_2_ on A549 cells exhibited a tail length of 2.05 ± 0.37, 93.43 ± 5.36, 73.83 ± 8.9, 150.38 ± 1.67, and 25.3 ± 6.96 (Table 2) (Figure 5(b)) and the OTM of 0.43 ± 0.07, 51.55 ± 5.0, 28.81 ± 4.94, 67.07 ± 5.98, and 9.51 ± 3.49 (Table 2) (Figure 5(c)), respectively.

The article "Cytotoxicity and Genotoxicity of Biogenic Silver Nanoparticles in A549 and BEAS-2B Cell Lines" was published in 2022. Journal: Bioinorg Chem Appl.

Conversely, all treatments (AgNPs-GA, Cisplatin alone, AgNPs-GA + Cisplatin, and H_2_O_2_) against BEAS-2B cells generated a significant or maximum DNA damage (Class 4 DNA damage) (Figure 4(b)) with the percentage of DNA in the tail values of 90.27 ± 2.0, 63.79 ± 3.01, 64.88 ± 2.55, and 85.86 ± 2.71, respectively, compared to the untreated (3.87 ± 2.63) (Table 2) (Figure 5(a)). The untreated and those treated with AgNPs-GA, Cisplatin, AgNPs-GA + Cisplatin, and H_2_O_2_ on BEAS-2B cells yielded a tail length of 3.87 ± 2.63, 86.32 ± 3.11, 160.07 ± 3.3, 160.85 ± 7.17, and 53.91 ± 9.95 (Table 2) (Figure 5(b)) and OTM of 0.7 ± 0.29, 49.19 ± 1.99, 78.49 ± 0.8, 80.9 ± 5.55, and 27.63 ± 4.6 (Table 2) (Figure 5(c)), respectively. The effects of AgNPs-GA are genotoxic, which causes harm to both A549 and BEAS-2B cells.

### 3.5. Mechanism of Apoptosis by 4′,6-Diamidino-2-Phenylindole (DAPI) and Acridine Orange (AO)/Propidium Iodide (PI) Double Staining

The mechanism of apoptosis was further investigated by DAPI and AO/PI double staining. Untreated cells in Figures 6(a) and 6(b) showed a normal smooth nuclear membrane, normal organelle structure, and intact cell membrane. However, the treatment with AgNPs-GA, Cisplatin, and AgNPs-GA + Cisplatin on both A549 and BEAS-2B cells changes the cell morphologies to cause cell shrinkage, nuclear chromatin condensation, nuclear chromatin fragmentation, and membrane blebbing. Damaged DNA in the nucleus exhibited a fluorescent blue colour. Besides that, the morphological change was also detected using an inverted microscope revealing damage to the cell membrane, shrinking of the cell population, and damage to the cell membrane of A549 and BEAS-2B cells (see Figures 6(a) (a) and 6(b) (a), respectively). However, the negative control cell displayed a completely intact morphology.

The results presented in Figures 6 and 7 reveal that the untreated cells (C-i) have healthy intact nuclei that are green and marked as no apoptosis. The observed effects were the appearance of chromatin condensation and fragmentation after 24 hours in cells treated with IC_50_ of AgNPs-GA (C-ii), Cisplatin (C-iii), and AgNPs-GA + Cisplatin (C-iv) indicating early apoptosis. Additionally, late-stage apoptosis was represented by the presence of orange membrane blebbing with an absence of cell necrosis. AgNPs-GA and Cisplatin have been shown to induce apoptosis in A549 and BEAS-2B cells, which is thought to be associated with increased levels of stress, DNA damage, and cell death.

### 3.6. Intracellular Silver Ion (Ag^+^) Concentration

The total silver content in the digested cells was measured after 24 hours using inductively coupled plasma optical emission spectroscopy (ICP-OES) to determine the amount of silver present in the A549 and BEAS-2B cells. In Figure 8, the amount of intracellular Ag content in A549 and BEAS-2B cells was 0.035 ± 0.001 ppm and 0.024 ± .001 ppm, respectively. Compared to the control, Ag-loaded AgNPs-GA + Cisplatin treated A549 and BEAS-2B cells absorbed around 0.031 ppm and 0.039 ppm of Ag, respectively.

The article "Cytotoxicity and Genotoxicity of Biogenic Silver Nanoparticles in A549 and BEAS-2B Cell Lines" was published in 2022. Journal: Bioinorg Chem Appl.

### 3.7. AgNPs-GA Intracellular Uptake and Localisation

Transmission electron microscopy (TEM) imaging was utilised to discover intranuclear particle localisation in A549 and BEAS-2B cells after exposure to the respective IC_50_ of AgNPs-GA, Cisplatin, and AgNPs-GA + Cisplatin. Following 24 hours of exposure, AgNPs-GA were mainly found within membrane-bound cytosol structures. The electron micrographs images are illustrated in Figure 9. Both of the A549 and BEAS-2B cells showed the absence of any abnormalities (Figures 9(a) and 9(b)). In contrast, AgNPs-GA and AgNPs-GA + Cisplatin treated A549 cells (Figures 9(c) and 9(g)) and BEAS-2B cells (Figures 9(d) and 9(h)) showed the presence of AgNPs-GA in the lysosomes. This suggests that nanoparticles can enter the cells through endocytosis and penetrate freely through cell membrane or diffusion.

The presence of significant quantities of AgNPs-GA (Figures 9(c), 9(d), 9(g), and 9(h)) in the cytoplasm supports the theory of direct uptake without the involvement of endosomes. Small numbers of nanoparticles are thought to help cells to survive longer; however, the presence of AgNPs-GA was detected in the nucleus (Figure 9(h)) and mitochondria (Figure 9(d)). Cisplatin exposure triggered many mitochondria cristae in both A549 and BEAS-2B cells (Figures 9(e) and 9(f)). Nuclear chromatin condensation observed with a nuclear membrane dilatation (Figures 9(e) and 9(h)) suggests the evidence of both apoptotic and necrotic/necroptotic cell morphology. Furthermore, in Figure 9(g), more vesicles are present in A549 cells treated with AgNPs-GA + Cisplatin. Cisplatin treated BEAS-2B cells showed a prominent cytoplasmic vacuole (Figure 8(f)).

## 4. Discussion

### 4.1. Biosynthesis of Silver Nanoparticles Mediated *G. atroviridis* Leaves Extract

In the previous study [36], we report the process of biogenic silver nanoparticles synthesis by using *G. atroviridis* leaf extract. The properties such as its size, shape, composition, and structural framework were confirmed by using UV-visible spectroscopy, scanning electron microscopy, transmission electron microscopy (TEM), dynamic light scattering, and X-ray diffraction analyses. Based upon this characterization, the size of AgNPs-GA was found in the range of 5–30 nm, whilst the shape was spherical with face-centered-cubic crystal structure. Further, FTIR data revealed that phenolic compounds were involved in the reduction of Ag^+^ into AgNPs-GA and could be responsible for the capping and stability of the AgNPs-GA [36]. The formation of AgNPs-GA can be observed as early as 24 h, evidenced by the appearance of brownish yellow colour after a short span of contact of Leaf-GA with silver nitrate salt (AgNO_3_) (Figure 1). This green synthesis technique involves reduction reaction as proposed by [45]:

(3) $$\begin{array}{c} {\text{Ag}}^{+}{\text{NO}}_{3}^{-}+\text{Plant molecule}\left(\text{OH},\text{C}=\text{H},\text{ etc}.\right)⟶{\text{Ag}}^{0}\text{nanoparticles .} \end{array}$$

Besides phytochemicals which act as reducing agent, the formation of AgNPs could also be derived through electrostatic interactions between the Ag^+^ ions and proteins found in plant material extract. The binding between these proteins with Ag^+^ ions could be via free amino or carboxyl groups [46]. These proteins are capable of reducing the silver ions causing structural changes and formation of silver nuclei that subsequently lead to the formation of AgNPs (Ag^0^) [45].

The article "Cytotoxicity and Genotoxicity of Biogenic Silver Nanoparticles in A549 and BEAS-2B Cell Lines" was published in 2022. Journal: Bioinorg Chem Appl.

### 4.2. In Vitro Assessment of AgNPs-GA, Leaf-GA, AgNO_3_, and AgNPs (Commercial) Toxicity on A549 and BEAS-2B Cell Viability

*G. atroviridis* of the Clusiaceae family is an annual plant and is found mostly in the humid tropics including Peninsular Malaysia and Sumatra [47, 48], possessing branched, erect, and pale yellow sap produced on the stems. The leaves are dark green, long, and narrow with a pointed tip and upturned edges, which are being used in folkloric medicine as pre- and postpartum medication [34, 48]. In the present study, the cytotoxicity of *G. atroviridis* leaf (Leaf-GA) was evaluated and compared with the efficacy of its silver nanoparticle form (AgNPs-GA). A weak cytotoxic activity was found when A549 and BEAS-2B cells were treated with Leaf-GA at concentration between 15.6 and 1000 *μ*g/mL (Figures 2(a) (ii) and 2(b) (ii)). Due to this, large doses of Leaf-GA were needed to suppress the cells. The IC_50_ values of Leaf-GA to inhibit 50% cell proliferation of A549 and BEAS-2B cells were determined to be 71–350 *μ*g/mL and 76–264 *μ*g/mL, respectively (Table 1). Interestingly, this study discovered that the biogenic silver nanoparticles from *G. atroviridis* leaf (AgNPs-GA) exhibit pronounced cytotoxic potential, with IC_50_ values of 20–31 *μ*g/mL and 12–42 *μ*g/mL in A549 and BEAS-2B cells, respectively (Table 1). In our previous study, *in vitro* cytotoxicity of the AgNPs-GA was also evaluated against human breast cell lines including MCF-7, MCF-7/TAMR-1, and MCF-10A [36]. Interestingly, we found a significant decrease in cell viability of all tested cell lines after exposure to AgNPs-GA by following concentration and incubation period manners. In fact, the possible mode of action mediated by AgNPs-GA was also explored through quantification of apoptotic cells by flow cytometric analysis. The data suggested that the mechanism of apoptosis was involved in AgNPs-GA-mediated cell death of MCF-7, MCF-7/TAMR-1, and MCF-10A [36].

The article "Cytotoxicity and Genotoxicity of Biogenic Silver Nanoparticles in A549 and BEAS-2B Cell Lines" was published in 2022. Journal: Bioinorg Chem Appl.

The cytotoxicity of AgNP depends on various factors including its physicochemical properties such as size, shape, and concentration [49]. The authors had summarised some size-dependent studies of AgNPs on different cell lines and they further proposed that smaller particles induce greater toxicity. Besides particle size, the cytotoxic potential of AgNP may also be affected by its shape. For example, Stoehr et al. [50] reported that silver wires showed significant cytotoxic effect on A549 cells, whereas no effects were observed for the spherical particles. However, in this study, the spherical shape of AgNPs-GA demonstrated significant cytotoxic activity against A549 and BEAS-2B human lung cells. As mentioned previously, the cytotoxic potential of AgNP might depend on multiple factors rather than a single one. The Trojan horse effect might play a role in the toxicity mechanism of AgNPs-GA. According to the Trojan horse theory, smaller size of AgNP has the capability to penetrate the cell membrane which is followed by ionic silver (Ag^+^) release inside the cells [51, 52]. These ions are considered as toxic ions due to the fact that they can interact with cellular structures and biomolecules including DNA, mitochondria, and proteins. This, in turn, might interrupt the normal cell multiplication, modulate the cytotoxic parameters, and finally lead to cell death [53, 54].

Literally, the formation of reactive oxygen species (ROS) and damaging the cell membrane are the most widely accepted cytotoxic mechanisms mediated by AgNPs. The Ag^+^ ions can generate ROS and cause lipid peroxidation inside the cells [53]. This later causes damage to cellular equilibrium through reactivity mechanism of positively charged Ag^+^ ions with the negatively charged oxygen and nitrogen atoms in the important organelles like DNA, mitochondrion, and the thiol group presented in protein structures and enzymes [53, 55]. Changes in the intracellular atmosphere of the cells, including alterations in the redox environment and loss of plasma membrane lipid asymmetry, are important regulators of the progression to apoptosis [56, 57]. The authors agreed to accept the fact that high level of ROS could potentially activate the mechanism of apoptosis in cells. Several AgNPs have been reported to act as inducers of ROS generation and apoptosis [58, 59]. The effects of AgNPs-GA on ROS production and induction of apoptosis were discussed in the following subsection.

The article "Cytotoxicity and Genotoxicity of Biogenic Silver Nanoparticles in A549 and BEAS-2B Cell Lines" was published in 2022. Journal: Bioinorg Chem Appl.

### 4.3. Analysis of Reactive Oxygen Species (ROS) Generation

The CM-H2DCFH-DA assay was used to determine the potential of AgNPs-GA, Cisplatin, and AgNPs-GA + Cisplatin in inducing oxidative stress by measuring the intracellular ROS levels. After treatment, an increase in ROS formation was observed in A549 and BEAS-2B cells demonstrated by an increase of DCF fluorescence intensity (Figure 3). ROS is a normal metabolic byproduct, which is vital in cell signalling and cell homeostasis. An increase in the intracellular ROS concentrations following chemotherapeutic drug exposures may result in significant alterations in cell morphology, cell damage that ultimately causes cell death. The DCFH-DA fluorescent dye was used in this study to examine the intracellular ROS activity in both A549 and BEAS-2B cells. DCFH-DA is deacetylated in the cytoplasm to yield a fluorescent compound of dichlorofluorescein (DCF) by cellular esterases. In this step, DCF is reduced into a fluorescent molecule by the radicals such as peroxyl, hydroxyl, nitrate, carbonate, and alkoxyl (excitation at 530 nm, emission at 485 nm) [60]. ROS is classified as molecules or ions containing an electron pair, and being a free radical, ROS is extraordinarily active due to unpaired electrons. It is involved in cell signalling and promoting oxidative cell damage. Cellular glutathione that is produced in a minimal amount neutralises ROS and keeps the cellular function normal [61]. A similar finding was observed in 4TI cells whereby AgNPs generated 38.25 and 44.13 ROS arbitrary units at 25 and 50 *μ*g/ml concentrations, respectively [62]. Another research group also reported that biosynthesized AgNPs from *Salvia miltiorrhiza* cause ROS released in the prostate cancer cell line (LNcap) [63].

It should be noted that the production of ROS is increased in the presence of smaller AgNPs compared to the larger AgNPs. For instance, AgNPs-1 caused an increase in the fluorescence intensity after exposure compared to AgNPs-70. These findings demonstrate that the mitochondrial ROS generation was enhanced following size-dependent manner of AgNPs [64]. Apart from the size of AgNPs, generation of ROS is also influenced by the time of exposure and concentration of AgNPs [61, 65].

It is very important to recognize the fact that high levels of ROS are detrimental to both normal and cancer cells, as it can destruct proteins, lipids, and DNA present in the cells. This results in nuclear fragmentation, membrane blebbing, cytoplasmic condensation, cell shrinkage, and death, a process called apoptosis. Elevation of ROS production and apoptotic cell death were evidenced in the present study. The AO/PI microscopic results demonstrated signs of apoptosis and dead cells following AgNPs-GA exposure in both A549 and BEAS-2B cell lines. This is in agreement with a study by Ali [66] that reported a significant correlation among ROS production, apoptosis, and DNA damage induced by AgNPs in freshwater snail *Lymnea luteola* L.

The article "Cytotoxicity and Genotoxicity of Biogenic Silver Nanoparticles in A549 and BEAS-2B Cell Lines" was published in 2022. Journal: Bioinorg Chem Appl.

### 4.4. Analysis of DNA Damage Activity

DNA damage can be referred to as abnormality to DNA chemical structure that changes its coding properties. Based on the source of the insult, DNA damage can be classified into two types, namely, endogenous damage caused by ROS and exogenous damage caused by ultraviolet and other types of radiation [67]. The common types of DNA damage include double-strand breaks (DSBs) and single-strand breaks (SSBs) [68]. In the present study, Comet Assay analysis, also known as Single Cell Gel Electrophoresis (SCGE), was used to determine the amount of DNA damage in individual cells. The Comet Assay is known for its simplicity and rapid performance [43], its capability to detect DNA damage in a variety of cell types [37], requiring minimal number of cells [69], and providing both qualitative and quantifiable index to evaluate DNA damage [39]. The principle of this assay is based upon the ability of damaged DNA to migrate out of the cell under electrophoresis that results in appearing like a comet tail. On the contrary, the undamaged DNA remains within the cell membrane creating the comet head [70].

The result herewith showed that DNA damage detected by the Comet Assay was observed in both human lung cancer (A549) and noncancer (BEAS-2B) cells after 24 h exposure to AgNPs-GA (Figure 4). Similar to our result, Kim et al. [41] reported 190.43–761.72 *μ*g/ml of AgNPs causes DNA damage in BEAS-2B cells (the same cells used in our study). Our finding is also in accordance with that reported by Nymark et al. [71], where DNA in comet tail was induced after both the 4 h and 24 h exposure to AgNPs. It is well-versed that reactive oxygen species (ROS) can cause progressive oxidative damage. This can occur when ROS is overproduced which later causes severe damage to cellular macromolecules such as DNA. This hierarchical process normally ended up with cell death if neither could oxidative stress be detoxified nor could defective DNA be repaired [66, 72]. The aforementioned notion is consistent with the data in this study whereby AgNPs-GA, Cisplatin, and AgNPs-GA + Cisplatin resulted in ROS generation, DNA damage that ultimately led to a mechanism of cell death.

The article "Cytotoxicity and Genotoxicity of Biogenic Silver Nanoparticles in A549 and BEAS-2B Cell Lines" was published in 2022. Journal: Bioinorg Chem Appl.

### 4.5. Mechanism of Apoptosis by DAPI and Acridine Orange (AO)/Propidium Iodide (PI) Double Staining

Apoptosis is a type of programmed cell death that occurs as a defense mechanism when cells are damaged beyond repair [44]. Mechanism of apoptosis can be triggered by various factors internal or external to the cell. It is well-versed that disproportionate amount of ROS may lead to apoptosis activation in a variety of human cancer and healthy cells [73]. As abovementioned, an increase in ROS production was observed in both A549 and BEAS-2B cells following exposure to AgNPs-GA. Therefore, apoptosis assay by using double staining with acridine orange/propidium iodide (AO/PI) was carried out to evaluate the mode of cell death causes by AgNPs-GA in both cell lines. AO is a standard nucleic acid dye that can permeate both viable and dead cells which emits green fluorescence upon intercalation with double-stranded (ds) DNA. Apoptotic cell death is characterized by orange fluorescence and this occurs when AO binds to the single-stranded DNA as a result of chromatin condensation or fracture fragments of DNA [74]. In contrast, PI is not membrane-permeable; therefore it can only penetrate dead cells to generate red fluorescence. For this reason, PI was employed to detect necrotic dead cells which are commonly characterized by the rupture of cell membrane, cell lysis, and release of cellular components [75].

As shown in Figures 6(c)-(i) and 7(c)-(ii), the untreated cells displayed fluoresced green with an intact nucleus indicating the cells were viable and healthy. On the contrary, both A549 (Figure 6(c)-(ii)) and BEAS-2B (Figure 7(c)-(ii)) cells treated with AgNPs-GA displayed majority of cells were at late stage of apoptosis. Typical apoptotic mode of cell death including cells blebbing and leakage of plasma membrane could be observed clearly with yellow-orange colour nuclei. Besides, spacing between cells due to the cell shrinkage and cells becoming rounded in form and smaller in size were also observed on AO/PI stained cell's population. Similar observation was made in cells treated with AgNPs-GA + Cisplatin. However, neither cells exhibited red fluorescence. These results are in accordance with other studies that employed AO/PI double staining to distinguish mechanism of apoptosis in cell culture systems. These include studies on toxicity effect of chlorhexidine on human corneal epithelial cells [76] and anticancer properties of AgNPs from *Clinacanthus nutans* leaves against oral squamous cancer cells [77]. The aforementioned studies used AO/PI staining to assess cell membrane integrity and determination of mode of cell death.

The article "Cytotoxicity and Genotoxicity of Biogenic Silver Nanoparticles in A549 and BEAS-2B Cell Lines" was published in 2022. Journal: Bioinorg Chem Appl.

### 4.6. Intracellular Ag^+^ Concentration and AgNPs-GA Intracellular Uptake and Localisation

In this study, ICP-OES was used to quantify the concentration of Ag element in cells after exposure to AgNPs-GA. The results showed A549 cells contain the highest Ag content (0.035 ppm), whilst BEAS-2B cells contain 0.024 ppm (Figure 8). The findings herewith may provide a good evidence to support the involvement of direct AgNPs-GA particle effect as well as dissolved Ag ions (Ag^+^). Regarding direct particle effects, Chen et al. [78] have described the surface of AgNPs may participate in the Fenton-like reactions to produce toxic hydroxyl radicals and subsequently exhibit biocidal properties. Associating with reports about the effect of Ag^+^, binding of Ag^+^ to glutathione (GSH) could lead to oxidative stress such as ROS, in cells [79, 80]. Besides GSH, Ag^+^ is also capable of binding the thiol groups of a host proteins, thereby inducing the cells to release ferrous ion (Fe^2+^). This hierarchical process leads to ROS and hydroxyl radicals formation through the Fenton reaction [80].

The uptake mechanisms were addressed herewith by using transmission electron microscopy (TEM) analysis. TEM images can provide evidence of the uptake mechanisms, intracellular localisation, and agglomeration of AgNPs. As shown in Figure 9, the AgNPs-GA was taken up by lysosomes and distributed throughout the cytoplasm, nucleus, and mitochondria. Similar findings are also reported in [61] on BEAS-2B cells with 10 *μ*g/ml of AgNPs for 24 h, whereby all AgNPs were mainly localised within membrane-bound structures, such as lysosomes. The authors also described the uptake was a combination of active mechanisms including clathrin-mediated endocytosis, micropinocytosis, and phagocytosis. In another study, Pritz et al. [81] have described macropinocytosis as one of the uptake processes of nanoparticles by the cells. They showed localisation of silica nanoparticles inside of endosome and lysosomes. As similar observations as described herewith, localisation profiles of AgNPs in porcine kidney (Pk15) cells were identified within lysosomes and early endosomes. The observed endocytic trafficking of AgNPs in both BEAS-2B human normal lung cells and Pk15 normal mammalian kidney cells may raise public safety concerns about their possible penetration into organisms, their accumulation in cells, and possible toxic effects. Nonetheless, lysosomes are digestive organelles which possess essential roles in degrading and recycling cellular waste, intracellular pathogen destruction, and apoptosis [82–84]. Lysosomes have also been proposed to be involved in degrading AgNPs to the Ag^+^ ion in the acidic lysosomal environment, which could interfere in the electron transport chain [80, 85]. Taken together, our findings herewith suggest the toxicity effects of AgNPs-GA in A549 and BEAS-2B cells could be associated with the internalization of free toxic Ag^+^ or by degradation of AgNPs-GA in the endocytic-lysosomal system or could be even reflecting an enhancement in lysosomal formation for detoxification purposes.

The article "Cytotoxicity and Genotoxicity of Biogenic Silver Nanoparticles in A549 and BEAS-2B Cell Lines" was published in 2022. Journal: Bioinorg Chem Appl.

Taken together, the results described herein indicate that exposure to the biosynthesized AgNPs could induce ROS production, inhibition of cell growth, disruption to cell membrane, and DNA damage, which are predominant mechanisms leading to toxicity. In fact, both human lung cell models, namely, A549 and BEAS-2B cells used in this study, were found to be sensitive towards exposure to the biosynthesized AgNPs-GA. The aforesaid findings are in accordance to the other metallic nanoparticles that affect human lungs through inhalation route [86, 87]. These metallic nanoparticles are capable of inducing pulmonary diseases and even injuries in other tissues. This fact has raised concerns and uncertainties about the possible risks of biosynthesized nanoparticles to human health, which emphasizes the urgent necessity and continuous efforts to get insight into risk assessment and toxicity characterization.

## 5. Conclusions

This study addresses mechanisms of toxic action following exposure to AgNPs-GA in 2 different cell lines, namely, A549 and BEAS-2B. AgNPs-GA was found to exert cytotoxicity in both A549 and BEAS-2B by inhibiting 50% cell proliferation at 20–28 *µ*g/mL and 12–35 *µ*g/mL concentrations, respectively. This cytotoxic effect of AgNPs-GA is associated with the induction of apoptosis as a mode of cell death. TEM shows nuclear chromatin fragmentation and cytoplasmic vacuoles in treated cells. Our findings also indicate that oxidative stress is one of the major toxic mechanisms of AgNPs-GA, as evidenced by a significant increase in ROS formation in both cells. The TEM results further confirm AgNPs-GA toxicity is predominantly mediated by intracellular uptake and subsequent release of Ag ions. Chemical analysis by inductively coupled plasma atomic emission spectroscopy indicates the presence of cellular dose of silver (between 0.024 and 0.035 ppm) in A549 and BEAS-2B cells. As AgNPs-GA are very small nanoparticles, they have the capability to penetrate the cell wall of both A549 and BEAS-2B cells. We also found that endocytosis is a crucial mechanism underlying the cellular uptake of AgNPs-GA in both cell lines. Furthermore, it was found that AgNPs-GA are located mainly within endolysosomal structures. These toxic properties are also associated with single-strand breaks of DNA (level 4 DNA damage) in both A549 and BEAS-2B cells.  Figure 10 summarises the proposed mechanism of AgNPs-GA toxicity based on the experimental data obtained in this study. In conclusion, our findings herein provide new insights towards the understanding the biological impacts of AgNPs-GA, particularly in A549 and BEAS-2B human lung cells. These adverse cell reactions towards exposure to AgNPs-GA could be prevented by applying safe concentrations of AgNPs-GA before seeking an alternative to this nanoparticle. Nevertheless, it is highly needed for further assessments on systemic distribution and other possible risks caused by AgNPs-GA exposure to human.

The article "Cytotoxicity and Genotoxicity of Biogenic Silver Nanoparticles in A549 and BEAS-2B Cell Lines" was published in 2022. Journal: Bioinorg Chem Appl.

## Figures and Tables

**Figure 1:** (a). Biosynthesis of G. atroviridis: (a) leaf-GA of *G. atroviridis* leaves, (b) synthesis of AgNPs-GA at 24 hours, (c) synthesis of AgNPs-GA at 48 hours, and (d) synthesis of AgNPs-GA at 72 hours. (b) UV-visible spectrum of AgNPs synthesis using Leaf-GA: spectrum of (a) AgNO3, (b) Leaf-GA, (c) AgNPs-GA at 24 hours, (d) AgNPs-GA at 48 hours, and (e) AgNPs-GA at 72 hours.

**Figure 2:** Line graph for IC_50_ value determination of (i) AgNPs-GA, (ii) leaf-GA, (iii) AgNO_3_, (iv) AgNPs (commercial), and (v) Cisplatin treatments against A549 (a) cells and BEAS-2B cells (b) at 24 hours, 48 hours, and 72 hours. Statistical analysis was determined by using Student's *t*-test (*a* = ^*∗*^*p* < 0.05, *b* = ^*∗∗*^*p* < 0.01, *c* = ^*∗∗∗*^*p* < 0.001) compared to the untreated cells.

**Figure 3:** Measurement of ROS level in AgNPs-GA, Cisplatin, and combination of AgNPs-GA + Cisplatin treated A549 and BEAS-2B cells at 24 hours. DCF fluorescence intensity was expressed in terms of ROS production. Values are expressed as fold change compared to the control (untreated cells). The intensity of the cells in the control group was set to 1. Statistical analysis was determined by using Student's *t*-test (*a* = ^*∗*^*p* < 0.05, *b* = ^*∗∗*^*p* < 0.01, *c* = ^*∗∗∗*^*p* < 0.001) compared to the untreated cells.

**Figure 4:** DNA damage of A549 (a) and BEAS-2B (b) cells was observed under fluorescence microscopy at ×100 magnification after being induced by AgNPs-GA, Cisplatin, AgNPs-GA + Cisplatin, and H_2_O_2_ compared to the untreated cells (negative control).

**Figure 5:** DNA damage analysis. (a) Percentage of DNA in the tail, (b) tail length (px), and (c) OTM induced by AgNPs-GA, Cisplatin, AgNPs-GA + Cisplatin, and H_2_O_2_ on A549 and BEAS-2B cells at 24 h. Statistical analysis was determined using one-way ANOVA followed by a post hoc Turkey multiple comparison test. ^Ψ^*p* < 0.05, ^ΨΨ^*p* < 0.01, ^ΨΨΨ^*p* < 0.001 for AgNPs-GA + Cisplatin compared to AgNPs-GA; ^Ω^*p* < 0.01, ^ΩΩ^*p* < 0.01, ^ΩΩΩ^*p* < 0.01 for AgNPs-GA + Cisplatin compared to Cisplatin; *a* = ^*∗*^*p* < 0.05, *b* = ^*∗∗*^*p* < 0.01, *c* = ^*∗∗∗*^*p* < 0.001 compared to the untreated cells.

The article "Cytotoxicity and Genotoxicity of Biogenic Silver Nanoparticles in A549 and BEAS-2B Cell Lines" was published in 2022. Journal: Bioinorg Chem Appl.

**Figure 6:** Representative image of A549 cells. (a) Morphology by inverted microscopy at ×100 magnification, (b) DAPI analysis, (c) merged AO/PI staining showing the effect of (i) untreated, (ii) AgNPs-GA, (iii) Cisplatin, and (iv) AgNPs-GA + Cisplatin on A549 cells at 24 hours. Morphological features of apoptosis including membrane blebbing (blue arrows), nuclear chromatin condensation (red arrows), and nuclear chromatin fragmentation (orange arrows) are evident. The fluorescent blue in DAPI images represents nucleus damage. Yellow and orange merged AO/PI images indicate an early and late-stage apoptosis, respectively. Images were captured at ×400 magnification.

**Figure 7:** Representative image of BEAS-2B cells. (a) Morphology by inverted microscopy at ×100 magnification, (b) DAPI analysis, (c) merged AO/PI staining showing the effect of (i) untreated, (ii) AgNPs-GA, (iii) Cisplatin, and (iv) AgNPs-GA + Cisplatin on BEAS-2B cells at 24 hours. Morphological features of apoptosis including membrane blebbing (blue arrows), nuclear chromatin condensation (red arrows), and nuclear chromatin fragmentation (orange arrows) are evident. The fluorescent blue in DAPI images represents nucleus damage. Yellow and orange merged AO/PI images indicate an early and late-stage apoptosis, respectively. Images were captured at ×400 magnification.

**Figure 8:** Measurement of intracellular Ag^+^ concentration (ppm) in AgNPs-GA, Cisplatin, and AgNPs-GA + Cisplatin treated A549 and BEAS-2B cells at 24 hours. Statistical analysis was determined using Student's *t*-test. ^*∗∗∗*^*p* < 0.001 compared to the untreated group.

**Figure 9:** Intracellular localisation of control and AgNPs-GA treated A549 and BEAS-2B cells at 24 hours by TEM. Control (untreated) cells show no morphological modifications (a, b). AgNPs-GA were taken up and deposited mainly within the membrane-bound structures (endocytosis). Magnified electron micrograph showing lysosomes containing AgNPs-GA (thick black arrow) (c(i), d(i), g(i), and h(i)). The presence of AgNPs-GA in the cytoplasm, nucleus, and mitochondria is indicated by a thin black, yellow, and thick blue arrow, respectively. The aggregation or cluster of AgNPs-GA is depicted by a thin red arrow (c(i)). Nuclear condensation and nuclear membrane dilatation (white arrow) (e and h). Phagosome (g). (N) Nucleus; Nu: Nucleolus; C: Cytoplasm; M: Mitochondria, P: Phagosome formation; L: Lysosomes; V: Vesicles. Magnification: a: ×2500; b: ×2500; c: ×4000, c(i): ×10000; (d) ×2000, d(i): ×6300; (e) ×4000, e(i): ×8000; (f) ×2000, f(i): ×5000; (g) ×5000, g(i): ×10000; (h) ×2000, h(i): 5000.

The article "Cytotoxicity and Genotoxicity of Biogenic Silver Nanoparticles in A549 and BEAS-2B Cell Lines" was published in 2022. Journal: Bioinorg Chem Appl.

**Figure 10:** Schematic diagram of the proposed mechanism of AgNPs-GA toxicity based on the experimental data obtained in this study.

**Table 1:** Summary of the AgNPs-GA, Leaf-GA, AgNO_3_, AgNPs (commercial), and Cisplatin average IC_50_ profiles against A549 and BEAS-2B cell lines and the SI.

Treatments	Time-point (h)	A549 cells (mean ± SD)	BEAS-2B cells (mean ± SD)	Selectivity index (SI)
AgNPs-GA	24	28.41 ± 2.54	35.47 ± 7.45	1.25
	48	28.76 ± 3.04	32.47 ± 7.85	1.13
	72	20.5 ± 2.66	12.13 ± 4.25	0.59

Leaf-GA	24	340.85 ± 8.13	255.13 ± 9.13	0.75
	48	154.06 ± 6.27	139.26 ± 6.35	0.90
	72	67.69 ± 4.06	68.24 ± 8.77	1.01

AgNO_3_	24	36 ± 0.01	16 ± 0.03	0.44
	48	31 ± 0.01	15 ± 0.02	0.48
	72	32 ± 0.05	14 ± 0.02	0.44

AgNPs (commercial)	24	1000 ± 0.01	735.68 ± 9.74	0.74
	48	539.15 ± 9.50	220.55 ± 7.79	0.41
	72	253.14 ± 3.37	153.73 ± 4.11	0.60

Cisplatin	24	52.48 ± 7.92	69.18 ± 1.75	1.32
	48	19.05 ± 3.19	31.62 ± 3.27	1.66
	72	17.48 ± 0.60	18.84 ± 0.13	1.08

**Table 2:** DNA damage induced by AgNPs-GA, Cisplatin, AgNPs-GA + Cislatin, and H_2_O_2_ on A549 and BEAS-2B cells. Statistical analysis was determined using one-way ANOVA followed by a post hoc Turkey multiple comparison test. ^*∗*^*p* < 0.05, ^*∗∗*^*p* < 0.01, ^*∗∗*^*p* < 0.001 compared to the untreated cells.

Treatments	Cells	Tail length (px)	% DNA in tail	Olive tail moment
Untreated	A549	2.05 ± 0.37	2.98 ± 0.57	0.43 ± 0.07
	BEAS-2B	3.87 ± 2.63	4.44 ± 0.97	0.7 ± 0.29

AgNPs-GA	A549	93.43 ± 5.36	87.9 ± 3.96	51.55 ± 5.0
	BEAS-2B	86.32 ± 3.11	90.27 ± 2.0	49.19 ± 1.99

Cisplatin	A549	73.83 ± 8.9	48.26 ± 4.54	28.81 ± 4.94
	BEAS-2B	160.07 ± 3.3	63.79 ± 3.01	78.49 ± 0.8

AgNPs-GA + Cisplatin	A549	150.38 ± 1.67	59.2 ± 1.6	67.07 ± 5.98
	BEAS-2B	160.85 ± 7.17	64.88 ± 2.55	80.9 ± 5.55

H_2_O_2_	A549	25.3 ± 6.96	35.64 ± 9.31	9.51 ± 3.49
	BEAS-2B	53.91 ± 9.95	85.86 ± 2.71	27.63 ± 4.6

## Data Availability

The cytotoxicity, genotoxicity, intracellular reactive oxygen species (ROS), mechanism of apoptosis, and cellular uptake of AgNPs-GA data used to support the findings of this study are included within the article. The physicochemical characteristic of AgNPs-GA to support the findings of this study can be referred to at https://doi.org/10.3390/molecules25184332.
